The article "Influence of COVID-19 pandemic on stress levels of urologic patients" was published in 2021. Journal: Open Med (Wars).

# Influence of COVID-19 pandemic on stress levels of urologic patients

**DOI:** 10.1515/med-2021-0289

**Published:** 2021-08-25

**Authors:** Michele Del Zingaro, Giovanni Cochetti, Giuseppe Maiolino, Davide Stivalini, Giulia Manfredini, Angelica Tancredi, Graziano Felici, Sara Ciarletti, Gianluca Gaudio, Jacopo Adolfo Rossi de Vermandois, Ettore Mearini

**Affiliations:** Department of Surgical and Biomedical Sciences, Division of Urology Clinic, University of Perugia, Perugia, 06129, Italy; Department of Surgical and Biomedical Sciences, Division of Urology Clinic, University of Perugia, Piazzale Giorgio Menghini 1, Perugia, 06129, Italy

**Keywords:** COVID-1, PSS-4, stress levels, urologic patients, urologic surgery

## Abstract

**Introduction:**

Several studies have shown the consequences of COVID-19 pandemic on perceived stress of different populations, but none of them analyzed urological patients who underwent elective surgery.

**Methods:**

We enrolled prospectively patients who underwent elective surgery between March and October 2020. A survey on COVID-19 and the 4-item Perceived Stress Scale (PPS-4) questionnaire were administered at hospital admission. Demographic and medical history data were also collected. Uni- and multivariate analyses were performed to identify independent predictors of higher PSS-4 values (≥7).

**Results:**

A total of 200 patients were enrolled. Mean PSS-4 value resulted 6.04. Patients with PSS-4 value ≥7 resulted 43.5% (87/200). In multivariate analysis, PSS-4 value ≥7 was independently associated (*p* < 0.05) with female gender (OR 6.42), oncological disease (OR 2.87), high (>5 in a range between 0 and 10) fear of intrahospital transmission of SARS-CoV-2 infection (OR 4.75), history of bladder instillation (OR 0.26), and current smokers (OR 0.27)

**Conclusion:**

High PSS-4 values at hospital admission in urologic surgical patients are positively correlated with female gender, fear of intrahospital transmission of SARS-CoV-2 infection, and oncological disease. PSS-4 questionnaire could be useful to select patients for whom a preadmission counselling is necessary to improve the management of their high stress level.

## 1 Introduction

Coronavirus disease (COVID-19) pandemic led to health, social, and economic consequences that nobody could foresee. Since the beginning of the pandemic at January 2021, almost 2 million deaths and 85 million coronavirus cases were recorded. These high numbers were caused by the extreme infectiousness of COVID-19, the severity of respiratory illness (Severe Acute Respiratory Syndrome coronavirus 2, SARS-CoV-2), and the absence of effective treatments. Common causes of death from COVID are pneumonia and ARDS, but COVID-19-associated coagulopathy can cause various thromboembolic complications, especially in critically ill patients [1].

The article "Influence of COVID-19 pandemic on stress levels of urologic patients" was published in 2021. Journal: Open Med (Wars).

Italy is the second country for deaths in proportion to COVID-19 cases or population (observed case-fatality ratio 3.5%) [2]. Many governments applied community measures aimed at social distancing: Italian government applied a national lockdown during March-May 2020 and further regional lockdowns based on Rt (or transmission index) and the resources of regional health services. Prevalence of stress, anxiety, depression among the general population [3,4,5], and health care system workers [6,7,8] has predictably increased: Tan et al. reported among surgical providers 32.8, 30.8, 25.9, and 24.0% screened positive for depression, anxiety, stress, and Post-Traumatic Stress Disorder (PTSD), respectively [9]. Ongoing studies are investigating the different factors involved to reduce the impact of COVID-19 pandemic on mental health, Quality of Life (QoL), and stress levels in the different populations [10], but none of these studies has focused on the impact of COVID-19 pandemic on stress levels of urologic patients who underwent urological elective surgery. During pandemic, in many hospitals of Italy, a great number of surgical procedures, including urological ones, were suspended or deferred. Teoh et al. in a global survey on the impact of COVID-19 on urological services reported a delay of >8 week in 28% of outpatient clinics, 30% of outpatient investigations and procedures, and 31% of urological surgeries. Urological services for benign conditions were more affected than those for malignant conditions [11].

According to the current guidelines [12], it was necessary to create levels of priority based on the predicted risk of clinical harms (progression, metastasis, loss of organ function), considering the available resources at the same time. Oncological and surgical patients are highly vulnerable to elevated stress levels, leading to serious psychological problems [13,14]. Health and social stress reduce their QoL and the pandemic could be another source of stress due to the fear of intrahospital infections, the lack of family support, and difficulties in managing any complication that could require the admission to intensive care unit.

Our study was primarily designed to evaluate the perceived stress levels among urologic patients who underwent urological elective surgery during the COVID-19 pandemic at hospital admission. The second aim was to explore the variables associated with higher perceived stress levels to make specific management programs for patients in order to reduce the risk of developing or worsening symptoms of depression and anxiety during and after hospitalization.

The article "Influence of COVID-19 pandemic on stress levels of urologic patients" was published in 2021. Journal: Open Med (Wars).

## 2 Methods

We prospectively enrolled patients who underwent urological elective surgery between March and October 2020 at our tertiary referral hospital. We developed a specific protocol both to provide a safe surgery for patient and surgical staff: before hospital admission, the risk of COVID infection was assessed by a phone triage investigating history of travel to endemic areas, previous contacts with a COVID-19-positive subject, or COVID-19-like symptoms within the last 2 weeks. Moreover, a PCR assay for SARS-CoV-2 detection was carried out for each patient by a nasal swab within 48 h before surgery. To reduce the lack of family support and the feeling of loneliness, we also offered a PCR assay for only one informal caregiver assisting the patient during hospitalization. All the physicians as well as nurses of the Urology Clinic were tested by nasal swab every two weeks. Moreover, patients from Emergency Department could be admitted to our ward only if negative for PCR assay, while if positive or uncertain, they were admitted to a specific COVID-19 ward. Ward-specific COVID prevention techniques were explained to the patients in detail prior to the procedure and prior to filling out the surveys. Exclusion criteria of our study were any conditions that could interfere with the ability to provide informed consent (educational level inferior to primary school, mental disability, dementia) or could confound the study outcomes (severe untreated psychopathology, e.g., schizophrenia, use of antipsychotics, immunologic, cardiovascular, renal or hepatic severe diseases or age >85 years). Participants self-completed the Italian version of PSS-4 questionnaire at hospital admission. Cohen et al. in 1983 [15] designed the Perceived Stress Scale, a self-reported questionnaire to evaluate how each person considers “situations in their lives as stressful” during the last month. This psychometric tool to measure global perceived stress levels is now available in three different versions and the 4-item scale (PSS-4) is used for settings with short time available [16]. An Italian version of Perceived Stress Scale was evaluated by Scale Mondo et al. in 2019 [17]. We provided the PSS-4 Italian Version as Supplemental Material.

A survey on COVID-19 was also administered: it was composed of two rating scale questions (0–10), the first about the fear of intrahospital infection of SARS-CoV-2 and the second about the patient’s trust in PPE (Personal Protective Equipment); in the rating scale, zero indicated that the patient had no fear and no trust, whereas ten corresponded to great fear and complete trust, respectively. The survey included also two closed-ended questions about a previous positive SARS-CoV-2 test or a close contact with a positive subject from the beginning of the pandemic. Demographic and medical history data were also collected: gender, age, educational level, marital status, household type (patients living with partners, partners and sons, other family members, or alone), smoking and alcohol habits, regular use of anxiolytics (Benzodiazepines, BZDs) or antidepressant drugs, Age-Adjusted Charlson Comorbidity Index (AACCI), oncological or non-oncological disease, organ involved in the surgical procedure, months from diagnosis, number of previous surgical procedures, history of radiotherapy, chemotherapy or bladder instillations, and type of procedure planned for their disease (endoscopic, open surgery, laparoscopic, or robot-assisted).

The article "Influence of COVID-19 pandemic on stress levels of urologic patients" was published in 2021. Journal: Open Med (Wars).

In descriptive statistical analysis parametric variables are given as the mean ± standard deviation (SD), nonparametric variables as their absolute and relative frequencies (*n*, %). In a first step, we performed *t*-student test and ANOVA to identify variables associated with different mean levels of PSS-4 score at admission. Based on literature, we considered a PSS-4 value ≥7 as marker of patients with significantly higher stress level in urologic patients who underwent elective surgery during COVID-19 pandemic. In second step of our analysis, in order to find independent predictors of PSS-4 values ≥7, we performed a univariate and multivariate logistic regression analysis. In the multivariate models, we included variables that resulted statistically significant in the univariate regression model. All reported *p* values are two-sided and statistical significance was set at 0.05. Statistical analysis was conducted using SPSS version 11.5 (SPSS, Chicago, Illinois). Local ethical committee approved the study protocol (PSSUROCHI v.1). All participants provided written informed consent and the study was conducted in accordance with the regulatory standards of the revised Declaration of Helsinki (2000).

## 3 Results

A total of 200 patients were enrolled, 186 men and 14 women. Two patients were excluded (one due to exceeded age limit and the other one due to mental disability). Baseline data of population study are fully reported in Tables 1 and 2. In our sample, the most common type of surgical procedure was endoscopic resection of bladder tumor (41%), followed by endoscopic resection of prostate and robot-assisted radical prostatectomy (36%), open and robot-assisted partial and radical nephrectomy (13%), and endoscopic resection of upper urinary tract urothelial carcinoma (8%). Table 3 showed results from survey on COVID-19 administered at hospital admission related with mean PSS-4 values. Mean value of PSS-4 at admission resulted 6.04 (±3.38). Different mean values of PSS-4 were significantly associated (*p* < 0.05) with age, gender, education level, marital status, household type, smoking status, benzodiazepines and antidepressant regular use, oncological vs non-oncological disease, organ-involved, history of surgical procedure, history of bladder instillations, type of procedure, and fear of intrahospital infection of SARS-CoV-2 (Tables 1–3). Patients with PSS-4 value ≥7 resulted 43.5% (*n* = 87/200). On multivariable analysis (Table 4), female gender (OR 6.42, 95% CI 1.08–39.1, *p* = 0.04), oncological disease (OR 2.87, 95% CI 1.07–7.68, *p* = 0.036), and a high (>5 in a range between 0 and 10) fear of transmission of SARS-CoV-2 infection (OR 4.75, 95% CI 2.06–10.9, *p* < 0.001) were positively associated with a PSS-4 value ≥7. History of bladder instillation (OR 0.26, 95% CI 0.12–0.56, *p* = 0.001) and current smokers (OR 0.27, 95% CI 0.10–0.72, *p* = 0.009) resulted, instead, negatively associated with PSS-4 ≥7 (Table 4).

The article "Influence of COVID-19 pandemic on stress levels of urologic patients" was published in 2021. Journal: Open Med (Wars).

**Table 1:** Demographic data and univariate analysis of mean values of PSS-4 at hospital admission

Variables		Patients *n* (%)	PSS-4 at admission (mean ± SD)	*p* value
Population study		200 (100)	6.04 ± 3.38	
Age (years)	20–40	12 (6)	4.17 ± 1.75	<0.01*
	41–60	30 (15)	6.43 ± 3.09	
	61–70	68 (34)	5.22 ± 3.11	
	71–85	90 (45)	6.78 ± 3.63	
Gender	Men	186 (93)	5.78 ± 3.16	<0.01*
	Women	14 (7)	9.50 ± 4.38	
Education level	Primary school	26 (13)	8.77 ± 3.04	<0.01*
	Secondary school	64 (32)	4.94 ± 3.52	
	High school	70 (35)	5.80 ± 2.76	
	Academic degree	40 (20)	6.45 ± 3.44	
Marital status	Single	8 (4)	2.00 ± 2.14	<0.01*
	With a partner	178 (89)	5.96 ± 3.07	
	Widowhood	14 (7)	9.43 ± 4.73	
Household type	Partner	110 (55)	5.81 ± 3.04	<0.01*
	Partner plus children	64 (32)	5.95 ± 3.03	
	Other family members	4 (2)	3.00 ± 2.00	
	Alone	22 (11)	8.00 ± 5.14	
Smoking status	Never or former smoker	164 (82)	6.39 ± 3.46	<0.01*
	Current smoker	36 (18)	4.44 ± 2.49	
Alcohol use	Not	130 (65)	6.29 ± 3.56	0.15
	Yes	70 (35)	5.57 ± 2.99	

PSS-4: 4-item perceived stress scale; *p < 0.05 with *t*-unparied test or ANOVA.

**Table 2:** Medical history data and univariate analysis of mean values of PSS-4 at hospital admission

Variables		Patients *n* (%)	PSS-4 at admission (mean ± SD)	*p* value
Population study		200 (100)	6.04 ± 3.38	
Age-adjusted Charlson comorbidity index	≤5	114 (57)	6.00 ± 3.35	0.85
	>5	86 (43)	6.09 ± 3.45	
BZDs use	Not	174 (87)	5.70 ± 3.22	<0.01*
	Yes	26 (13)	8.35 ± 3.59	
Antidepressants use	Not	196 (98)	5.93 ± 3.31	<0.01*
	Yes	4 (2)	11.50 ± 2.38	
Disease	Not oncological	32 (16)	4.75 ± 2.44	0.02*
	Oncological	168 (84)	6.29 ± 3.48	
Organ-involved	Bladder	82 (41)	6.22 ± 3.25	<0.01*
	Prostate	72 (36)	5.85 ± 2.84	
	Kidney	26 (13)	8.23 ± 4.26	
	Ureter or pelvicalyceal systems	16 (8)	3.06 ± 2.35	
	Testis	4 (2)	3.50 ± 2.38	
Months from diagnosis	≤5	86	5.66 ± 3.38	1.17
	>5	114	6.32 ± 3.37	
Number of previous surgical procedure	≤5	138	6.39 ± 3.33	0.03*
	>5	62	5.26 ± 3.40	
History of radiotherapy	Not	182	6.03 ± 3.48	0.89
	Yes	18	6.11 ± 2.25	
History of chemotherapy	Not	192	6.08 ± 3.40	0.38
	Yes	8	5.00 ± 2.83	
History of bladder instillations	Not	132	6.42 ± 3.41	0.03*
	Yes	68	5.31 ± 3.24	
Type of procedure	Open surgery	12	4.67 ± 3.37	0.00*
	Laparoscopic-assisted	4	4.75 ± 1.50	
	Endoscopic	126	5.56 ± 3.12	
	Robot-assisted	58	7.45 ± 3.65	

PSS-4: 4-item perceived stress scale; BZDs: benzodiazepines; *p < 0.05 with *t*-unparied test or ANOVA.

The article "Influence of COVID-19 pandemic on stress levels of urologic patients" was published in 2021. Journal: Open Med (Wars).

**Table 3:** Survey on COVID-19 and univariate analysis of mean values of PSS-4 at hospital admission

		Patients *n* (%)	PSS-4 at admission (mean ± SD)	*p* value
Previous positive test for SARS-CoV-2	Not	200	6.04 ± 3.38	—
	Yes	0	0 ± 0	
Close contact with people with positive test for SARS-CoV-2	Not	192	6.08 ± 3.42	0.38
	Yes	8	5.00 ± 2.14	
Fear of intrahospital infection of SARS-CoV-2 (range 0–10)	≤5	154	5.12 ± 2.82	0.000*
	>5	46	9.13 ± 3.30	
Trust in PPE (range 0–10)	≤5	76	6.11 ± 3.66	0.83
	>5	124	6.00 ± 3.21	

PPE: personal protective equipment. *p < 0.05 with *t*-unparied test or ANOVA.

**Table 4:** Univariate and multivariate logistic regression analysis of clinical factors in predicting PSS-4 ≥7 (*n* = 87/200–43.5%)

	Univariate analysis			Multivariate analysis		
	OR	95% CI	*p* value	OR	95% CI	*p* value
Age classes						
20–70	Reference					
71–85	2.26	1.28–4.01	0.005*	1.79	0.89–3.57	0.09
Gender						
Male	Reference					
Female	5.30	1.43–19.66	0.012*	6.42	1.08–39.1	0.04*
Level of education						
Academic degree	Reference					
Primary school	1.89	0.68–5.22	0.221	—	—	—
Secondary school	0.49	0.22–1.09	0.083	—	—	—
High school	0.71	0.32–1.54	0.385	—	—	—
Marital status						
Widowhood	Reference					
Single	0.00	—	0.99	—	—	—
With a partner	0.30	0.092–1.00	0.052	—	—	—
Household type						
Partner	Reference					
Partner plus children	0.92	0.49–1.71	0.79	—	—	—
Other family members	0.00	—	0.99	—	—	—
Alone	2.34	0.91–6.05	0.78	—	—	—
Smoking status						
Never or former smoker	Reference					
Current smoker	0.31	0.13–0.71	0.006*	0.27	0.10–0.72	0.009*
BZD use						
No	Reference					
Yes	2.32	0.99–5.41	0.051	—	—	—
Antidepressants use						
No	Reference					
Yes	0.00	—	0.99	—	—	—
Number of previous surgical procedure						
≤5	Reference					
>5	1.33	0.72–2.45	0.36	—	—	—
Disease						
Not oncological	Reference					
Oncological	2.66	1.13–6.26	0.025*	2.87	1.07–7.68	0.036*
Organ-involved						
Testis	Reference					
Bladder	2.85	0.28–28.61	0.37	—	—	—
Prostate	2.02	0.20–20.41	0.55	—	—	—
Kidney	4.80	043–52.76	0.20	—	—	—
Ureter or pelvicalyceal system	0.20	0.01–4.17	0.29	—	—	—
History of bladder instillation						
Not	Reference					
Yes	2.02	1.10–3.74	0.02*	0.26	0.12–0.56	0.001*
Type of procedure						
Open surgery	Reference					
Laparoscopic-assisted	0.33	0.27–4.18	0.39	—	—	—
Endoscopic	0.61	0.18–2.01	0.42	—	—	—
Robot-assisted	1.23	0.35–4.27	0.74	—	—	—
Fear of intrahospital transmission of SARS-CoV-2 infection (1–10)						
≤5	Reference					
>5	7.27	3.34–15.8	<0.001*	4.75	2.06–10.9	<0.001*

OR: odds radio; CI: confidence interval. Bold indicates that *p* < 0.05 on univariate and multivariate analysis.

The article "Influence of COVID-19 pandemic on stress levels of urologic patients" was published in 2021. Journal: Open Med (Wars).

## 4 Discussion

During global SARS-CoV-2 pandemic, patients waiting for urological surgery experienced the loneliness caused by social distancing measures, the fear of disease progression due to the deferral of a great number of surgical procedures, the concern for intrahospital SARS-CoV-2 infection, and the absence of a family support as a result of visiting restrictions. For these reasons, mental and emotional state of patients waiting for urological surgery was radically changed by the pandemic.

In our study, mean PSS-4 score at admission resulted in greater than values as reported by the Spanish and French studies [18,19] and similar normative data from English sample reported by Warttig et al. [20] in general population. Our findings confirmed results related to general population as reported in other studies: different mean values of PSS-4 were significantly associated with age [18,20], gender [18,20], education level [18,19,21], smoking [22], and marital status [18]. Furthermore, in our study based on patients undergoing urology procedures new variables resulted that were significantly associated with different mean of PSS-4 score values: benzodiazepines and antidepressant regular use, type of disease (oncological vs benign disease), organ-involved, history of surgical procedure, history of bladder instillations, type of procedure, and fear of intrahospital infection of SARS-CoV-2. These new variables are probably related to the specific features of analyzed sample which differs from general population.

The perceived stress levels of patients waiting for surgery are higher than general population beyond COVID-19 outbreak [23] and another additional source of stress could cause disastrous consequences. The exposure to stress has long-term health effects including increased risk of physical and mental disorders, impaired cognitive function, and reduced productivity and absenteeism from work [24]. In surgical patients, for example, psychological stress has been shown to impair wound healing: Broadbent et al. reported that a brief relaxation intervention prior to surgery can reduce stress and improve the wound healing response in surgical patients [25]. Psychological characteristics widely influence the pathophysiological mechanisms underlying the neuroendocrine and inflammatory response to surgical stress, potentially interfering with surgical outcomes [26]. For these reasons, it is important to identify risk factors for high stress levels to prevent and reduce the impact of stressors.

The article "Influence of COVID-19 pandemic on stress levels of urologic patients" was published in 2021. Journal: Open Med (Wars).

PSS-4 is a psychometric tool that is not used for diagnosis, but to compare an individual score to normative value. In literature, there are no studies which analyzed the average value of PSS-4 among Italian people or patients undergoing urology procedures. For this reason, in our study we considered values related to European population: a recent Spanish study [18] analyzed a sample of 37,451 people taken from the general population (the largest sample analyzed in literature), showing a total average value of PSS-4 of 5.43 (average male value: 5.25; average female value: 5.60). Lesage et al. based on French population reported a total average value of 5.40 [19]. Warttig et al. provided normative value from English sample (*n* = 1,484) that reported a mean value of PSS-4 of 6.11 [20]. We arbitrarily considered a PSS-4 value ≥7 as marker of patients with significantly higher stress level and we performed a multivariate analysis in order to find independent predictors for PSS-4 values ≥7. PSS-4 ≥7 resulted positively correlated with female gender, oncological disease, and a high (>5 in a range between 0 and 10) fear of intrahospital transmission of SARS-CoV-2 infection, while negatively correlated with history of bladder instillation and current smokers.

Female gender is a well-established risk factor for high stress levels: Cohen and Williamson’s original PSS-4 study in 1988 showed statistically significant differences in the scores between men and women, with women reporting the highest scores [27]. These findings have been supported by later studies [20,28]. Two hypotheses to explain these differences have been proposed in literature: a differential vulnerability even when the stressors are identical or a differential exposure to higher levels of stressors than men. Moreover, gender is associated with a different perception of a particular situation as stressful and with subsequent coping methods [29].

Oncological patients are vulnerable to distressed psychological states. The prevalence of psychological distress is correlated to type of cancer, time since diagnosis, degree of physical and social role impairment, amount of pain, prognosis, and other variables [30].

The article "Influence of COVID-19 pandemic on stress levels of urologic patients" was published in 2021. Journal: Open Med (Wars).

Our study showed that higher fear of intrahospital transmission of SARS-CoV-2 infection is a further risk factor for high stress levels. This finding is a new stressor factor related to COVID-19 pandemic and surgery urologic patients. Our results are in line with Campi et al. that reported of 332 patients scheduled for elective urological procedures, 47.9% would have deferred the planned intervention and 80–87% of them answered for more than 6 months. These answers were influenced by patient’s age, American Society of Anesthesiologists, and underlying urological condition. Finally, 182 (54.8%) patients considered the risk of COVID-19 potentially more harmful than the risk of delaying surgery [31].

About the negative correlation between high stress levels (PSS-4 ≥7) and history of bladders instillations, we hypothesize that patients who underwent bladder instillations showed a lower stress levels for two reasons: (1) this subgroup, including mostly patients with low-risk noninvasive bladder cancer, is familiar with hospital setting due to history of recurrent transurethral resection of bladder tumor; and (2) they believed that bladder instillations performed in outpatient setting both reduce the progression and recurrence risk, preventing the risk of hospitalization. Schmidt and colleagues [32] reported a statistically significant improvement in mental health composite scores of short form-36 physical and mental health questionnaire after transurethral resection and intravesical mitomycin C compared with transurethral resection alone.

Smoking has been already correlated with lower stress levels in other reports [33], but there are many complex interactions between stress and smoking onset, maintenance, and relapse [34].

The limitations of our study are the small sample, the absence of validation of PSS-4 in hospital admission setting, and the lack of normative value in this setting. Another limitation is the absence of other psychological instruments to measure the stress levels and to compare them to PSS-4 results. Regarding survey on COVID-19 used in our study, a limitation is a possible misunderstanding about trust in PPE and fear of intrahospital infection of SARS-CoV-2 that represent opposite ends of the trust and fear spectrum.

We concluded that PSS-4, a simple and short questionnaire, administered at hospital admission has proven to be correlated to general population stress-related factors (age, educational level, smoking status, and others), to urologic patients stress-related factors (oncological vs non-oncological disease, organ-involved, history of surgical procedure, history of bladder instillations, type of procedure), and to COVID-19 stress-related variables (fear of intrahospital transmission). This tool could be used to screen patients before hospital admission during COVID-19 pandemic, identifying those with increased risk of high and significant stress level. This risk stratification may be useful to select patients who could benefit from a prehospital admission counselling in order to improve the management of their high stress level with specific strategies [24].
